The article "Design and Analysis of Adolescent Physical Health Monitoring System under the Background of Internet of Things and 5G" was retracted in 2023. Reasons: signs of a paper mill; suspected computer-generated content; unreliable results or conclusions; lack of ethics approval or compliance.

# Design and Analysis of Adolescent Physical Health Monitoring System under the Background of Internet of Things and 5G

**DOI:** 10.1155/2021/5208976

**Published:** 2021-11-15

**Authors:** Zhi Chen

**Affiliations:** School of Physical Education, Anhui Polytechnic University, Wuhu 241000, China

## Abstract

In recent years, with the rapid development of network communication, 5G technology has brought about higher network speed and more communication requirements. Internet of Things technology has been widely used in many fields. Therefore, this paper realizes the physical health monitoring system under the Internet of Things and 5G communication technology to detect the physical health of teenagers in real time. Based on the in-depth analysis of the theoretical research and application status of the healthy Internet of Things at home and abroad, this paper first studies the theories and methods of teenagers' physical health information collection, collects human body temperature and movement steps, respectively, through wearable devices based on RFID anticollision algorithm, and further estimates human health and movement. The prototype system of the adolescent physical health monitoring system is realized. The system is divided into the terminal node and client information management system: (1) The terminal node is divided into information collection node and information collection node. The hardware circuit of the collection node mainly includes a microcontroller module, a sensor module, and a power circuit, and the collection node mainly includes a microcontroller module, a serial port module, and a power circuit. (2) The client information management system is divided into PC end and the mobile end. The PC end uses asp.net and SQL Server technology to design the database and user interface, and the mobile end uses WeChat public platform for development and design.

## 1. Introduction

In recent years, the physical health level of teenagers in China has been declining continuously. Many authoritative investigations have pointed out that the hidden problem behind it is that the current physical education curriculum is a mere formality and the supervision of physical education tests is insufficient, which has caused all sectors of society to pay close attention to the physical health of teenagers [1]. The RFID electronic tag can be used in the youth sports test process to bind the youth identity [2] and ensure the authenticity of sports test data. Therefore, based on the grim situation of students' physical health and the good development prospect of wearable devices, combining wearable technology, 5G communication technology, and RFID identification technology, a physical health monitoring system is designed, which integrates various physical data collection and effective identity matching functions. Teenagers' identities are matched through RFID chips, physical data generated in teenagers' exercise process and centralized test in real time through sensors are collected, and finally data transmission with clients is realized through 5G communication function [3], so as to achieve the purpose of monitoring teenagers' physical health and improving their physical fitness.

The article "Design and Analysis of Adolescent Physical Health Monitoring System under the Background of Internet of Things and 5G" was retracted in 2023. Reasons: signs of a paper mill; suspected computer-generated content; unreliable results or conclusions; lack of ethics approval or compliance.

The 5th-generation mobile communication technology is a new generation of broadband mobile communication technology with the characteristics of high speed, low delay, and large connection. It is the network infrastructure to realize man-machine interconnection. 5G will gradually pierce all industries and sectors of the economy and society and become a key new infrastructure to support the digitalization, networking, and intelligent transformation of the economy and society. The Internet of Things is the Internet, the traditional telecommunications network, and other information carriers so that all ordinary objects can perform independent functions to achieve an interconnection network. The Internet of Things technology is based on 5G and core of the Internet technology, and the completion of the information exchange and communication process is also based on Internet technology. Communication technology is closely related to the Internet of Things, and technologies such as mass terminal connection and real-time control in the Internet of Things cannot do without high-speed communication technology. 5G stimulates the development of the Internet of Things, and the Internet of Things is the prelude and foundation of the commercial use of 5G. 5G and the Internet of Things are complementary to each other, and the two interact to jointly benefit the development of human society. The realization of 5G will not only bring about profound influence to the Internet of Things but also greatly promote the development of a social economy. It will create great value in smart agriculture, smart logistics, smart home, Internet of vehicles, smart city, and other fields.

With the rapid development of science and technology and communication, all fields are intertwined. The rise of 5G network has also brought about many new technology applications, and the development of Internet, medical care, and 5G has begun. We propose a 5G-assisted intelligent sports and healthcare solution assisted by IoT, which needs equipment, energy efficiency, and necessary security support, which is a difficult point [4]. Through analysis, it can be seen that, to solve this challenge, relevant literature should be presented in the structure of 5G smart medicine. In addition, intelligent sports and medical care systems are also the keys to successfully deploy 5G. For a long time, society and the country have paid great attention to the health problems of teenagers. We use various programs to educate them about health and encourage them to have an active lifestyle to reduce health risks, such as questionnaires and game-based programs. However, due to the lack of professional healthcare personnel to verify it, these methods cannot achieve satisfactory results. To this end, we analyzed the advantages of the application and the recognition of teenagers and then found the obstacles encountered by some teenagers in the process of using it through sample survey, as well as the relationship between the evaluation obtained by using the Fisher test to answer the questionnaire and adopting a healthier diet and exercise practice. Finally, I learned that mobile applications are popular, and, to some extent, their daily eating habits have improved [5]. Smart wearable devices have become popular in people's lives and play an active role in monitoring adolescents' health. They can obtain the data of the wearer, but the analysis of the data is not deep enough, and the value extraction is not high. On the existing basis, we developed a machine-learning-based fitness evaluation model for teenagers' wearable running monitoring, which was combined with parameter optimization to establish a fitness evaluation model. Firstly, photo plethysmography (PPG) signals of adolescents' activities are collected by smart bands, and then the signals are converted into physiological data such as heart rate. After the key features are extracted by the feature engineering module, high-grade schemes are selected by sequence forward search (PC-ISR-SFS). Finally, an extreme gradient boosting (XGBoost) algorithm is used to classify adolescents' health levels. After verification, the model has higher evaluation accuracy, which replaces the traditional evaluation model to a certain extent and provides a more advanced model for the evaluation scheme of teenagers' physical health [6].

The article "Design and Analysis of Adolescent Physical Health Monitoring System under the Background of Internet of Things and 5G" was retracted in 2023. Reasons: signs of a paper mill; suspected computer-generated content; unreliable results or conclusions; lack of ethics approval or compliance.

While the network brings about great convenience to our life and work, it also has some bad influences to some extent. Social networks are becoming increasingly popular among teenagers, and most teenagers use online profiles and communication to reflect unhealthy behaviors in the world of social networks. On the Internet, we believe that teenagers use a variety of impression management strategies. To test this idea, we analyzed 5,851 posts. It can be seen that teenagers will show their health information in order to attract the attention of their peers or to show off, so we can judge that those unhealthy behaviors are more attractive than offline socializing [7]. The whole world has been paying attention to the physical health of teenagers for a long time, especially in the growth and development stage. The lack of exercise of teenagers will affect the premature degradation of their central nervous system and the deterioration of their physical fitness. Physical exercise for teenagers is very important. We can generally regulate and quantify the effect of exercise by monitoring real-time exercise and collecting data. Aiming at the monitoring and quantitative evaluation of data, we put forward a monitoring and evaluation method of sports training effect based on reinforcement learning (RL) and the Markov model. Compared with the traditional monitoring mechanism, this method can train them more efficiently, and the deviation rate of evaluation is very low [8]. By combining 5G and the Internet of Things, our proposed system can be used to detect the physical health information of teenagers in real time, and, according to the quantified health level and exercise amount, it can achieve the purpose of monitoring teenagers' physical health [8].

## 2. Research on RFID Anticollision Algorithm of Wearable Devices Based on Internet of Things

With the rapid development and wide application of the Internet of Things and 5G technology [9], wearable devices with built-in RFID electronic tags are gradually increasing. RFID electronic tags have a unique built-in ID code, so RFID anticollision algorithm is widely used in wearable devices [10].

### 2.1. RFID Anticollision Algorithm Principle Analysis

In the PA algorithm, after the tag in the recognizable range of the reader is activated, the identification information will be randomly sent to the reader. There may be two situations: complete collision or partial collision in the identification information of multiple tags [11]. When there is a collision, the tag will generate random waiting time, and then after the random waiting time ends, it will continue to send identification information to the reader until it is successfully identified. After the reader successfully identifies the tag information, it will send a response signal to the corresponding tag, and the corresponding tag will enter a dormant state. When all the tags are successfully identified, the algorithm ends. In the PA algorithm, the tags send data at random time, the sending time of multiple tags partially overlaps, and the data sent by tags interfere with each other; that is, there is partial conflict. Therefore, its throughput rate is extremely low, only 18.4%.

The article "Design and Analysis of Adolescent Physical Health Monitoring System under the Background of Internet of Things and 5G" was retracted in 2023. Reasons: signs of a paper mill; suspected computer-generated content; unreliable results or conclusions; lack of ethics approval or compliance.

In order to solve the partial collision phenomenon of the PA algorithm, the SA algorithm came into being.

### 2.2. Establishment and Design of Algorithm Model

In view of the shortcomings of existing algorithms, this chapter proposes a new RFID anticollision algorithm for monitoring adolescents' health.

#### 2.2.1. Basic Definitions

BEAD algorithm divides a frame into T time slots, defines the number of instantaneous slots as T, and defines the total number of identification object tags within the reader recognition range as M. Since the process of selecting time slots for tags is an independent selection process that is not related to the others, the matching identification process of tags and time slots is considered as multiple Bernoulli tests [12] because the matching identification process of tags and time slots has nothing to do with other tags; you can transform it into a mathematical problem of the binomial distribution.

The specific probability is expressed as

(1) $$\begin{array}{c} P\left(X=k\right)=C_{m}^{k}\cdot \left(\frac{1}{T}\right)\cdot {\left(1-\frac{1}{T}\right)}^{m-k}. \end{array}$$

If *k* ∈ [0, *m*] and *k* are rounded and *k* = 1, the probability of a successful time slot can be obtained according to the above formula; that is, the probability that only one label is selected in one-time slot is

(2) $$\begin{array}{c} P_{g}=P\left(X=1\right)=C_{m}^{1}\cdot {\left(\frac{1}{T}\right)}^{1}\cdot {\left(1-\frac{1}{T}\right)}^{m-1}=\frac{m}{T}\cdot {\left(1-\frac{1}{T}\right)}^{m-1}. \end{array}$$

By the same token, when *k* = 0,

(3) $$\begin{array}{c} P_{l}=P\left(X=0\right)=C_{m}^{0}\cdot {\left(\frac{1}{T}\right)}^{0}\cdot {\left(1-\frac{1}{T}\right)}^{m-0}={\left(1-\frac{1}{T}\right)}^{m}. \end{array}$$

When *k* ≥ 2, the probability of collision slot can be expressed by the principle that the sum of probabilities is 1:

(4) $$\begin{array}{c} P_{e}=p\left(X\geq 2\right)=1-P\left(X=1\right)-P\left(X=0\right). \end{array}$$

Under ideal conditions, the expectation of a specified successful time slot, the expectation of an idle time slot, and the expectation of a collision time slot are, respectively, expressed by *a*_*g*_^*T*,*m*^, *a*_*l*_^*T*,*m*^, and *a*_*e*_^*T*,*m*^; their mathematical expressions are as follows:

(5) $$\begin{array}{c} a_{g}^{T,m}=T\cdot P_{g}=m\cdot {\left(1-\frac{1}{T}\right)}^{m-1},\\ a_{l}^{T,m}=T\cdot P_{l}=T\cdot {\left(1-\frac{1}{T}\right)}^{m},\\ a_{e}^{T,m}=T\cdot P_{e}=T-a_{g}^{T,m}-a_{l}^{T,m}. \end{array}$$

Consider that the system throughput rate is *S*_*RFI*  *D*_, and the formula is

(6) $$\begin{array}{c} S_{RFID}=\frac{a_{g}^{T,m}}{T}=\frac{m}{T}\cdot {\left(1-\frac{1}{T}\right)}^{m-1}. \end{array}$$

Deriving formula (6) leads to

(7) $$\begin{array}{c} \frac{ds}{dm}=\frac{1}{T}\cdot {\left(1-\frac{1}{T}\right)}^{m-1}+\frac{m}{T}\cdot {\left(1-\frac{1}{T}\right)}^{m-1}In\left(1-\frac{1}{T}\right). \end{array}$$

By finding the extreme value of equation (7), the functional relationship between the number of time slots and the number of labels can be obtained as follows:

(8) $$\begin{array}{c} \frac{ds}{dm}=\frac{1}{T}\cdot {\left(1-\frac{1}{T}\right)}^{m-1}+\frac{m}{T}\cdot {\left(1-\frac{1}{T}\right)}^{m-1}In\left(1-\frac{1}{T}\right). \end{array}$$

Equation (8) shows that if the number of time slots that the system can allocate is equal to the number of tags and if the number of tags is greater than 1, the throughput of the system reaches the extreme value. In addition, if all time slots are idle or if the collision does not have a flag identifying all responses, the throughput rate is a minimum value of 0. During one identification, if all tags are normally identified, the throughput rate reaches a maximum of 1.

The article "Design and Analysis of Adolescent Physical Health Monitoring System under the Background of Internet of Things and 5G" was retracted in 2023. Reasons: signs of a paper mill; suspected computer-generated content; unreliable results or conclusions; lack of ethics approval or compliance.

#### 2.2.2. Isoregional Groupings

All the labels within the recognition range of the card reader are grouped based on the idea of equal-area division, that is, sector grouping centered on the card reader. The purpose is to improve the recognition efficiency of the system by identifying each tag group. The structure of the equal-area packet is shown in Figure 1.

In a wireless communication system, since the channel varies with time, it is necessary to consider the path loss due to the distance between the tag and the reader. In the wireless channel, the average received power of the system is

(9) $$\begin{array}{c} P_{r}=P_{t}+10\lambda \mathrm{lg}\frac{d}{d_{0}}. \end{array}$$

#### 2.2.3. Estimated Number of Labels

The numbers of successful time slots, idle time slots, and collision time slots are set to *T*_*g*_, *T*_*l*_, and *T*_*e*_, respectively. Assuming that there is a linear functional relationship between the total number of labels to be identified and the number of collision slots after *n* rounds of query, the prediction formula of the number of labels in *n* + 1 rounds is

(10) $$\begin{array}{c} P_{r}=P_{t}+10\lambda \mathrm{lg}\frac{d}{d_{0}}. \end{array}$$

Therefore, when the estimation of the tag number of the (*n* + 1) round is started, the estimated waiting tag number of the current frame is calculated using the DFSAC-II algorithm, and the prediction result of the *n*th round is adjusted:

(11) $$\begin{array}{c} m_{adjust\left(n+1\right)}=2.3922\cdot T_{e\left(n+1\right)}. \end{array}$$

Then, the theoretical error value can be obtained by subtracting the prediction result of the *n*th round from the adjustment result of the *n* + *l* round:

(12) $$\begin{array}{c} \varepsilon =m_{predict\left(n+1\right)}-m_{a\;dj\;ust\left(n+1\right)}=\xi T_{e\left(n\right)}-2.3922T_{e\left(n+1\right)}. \end{array}$$

In order to obtain the minimum error, the minimum value is obtained by deriving the square of the theoretical error value concerning *ξ*:

(13) $$\begin{array}{c} \partial \frac{\varepsilon^{2}}{k}=2\left[\xi T_{e\left(n\right)}-2.3922T_{e\left(n+1\right)}\right]\cdot T_{e\left(n\right)}. \end{array}$$

If formula (13) is 0, the dynamic prediction weight of the label estimation is

(14) $$\begin{array}{c} \xi =\frac{2.3922T_{e\left(n+1\right)}}{T_{e\left(n\right)}}. \end{array}$$

Since the number of collision slots in the next round cannot be obtained in advance in the actual execution of the algorithm, the formula is modified in association, and the dynamic prediction value can be obtained by substituting the number of slots in this round and the number of slots in the previous round into the above equation. Therefore, *ξ* is

(15) $$\begin{array}{c} \xi =\frac{2.3922T_{e\left(n\right)}}{T_{e\left(n-1\right)}}. \end{array}$$

Substituting *ξ* into equation (10), the number of predicted labels in the next round can be as follows:

(16) $$\begin{array}{c} m=\frac{2.3922{\left[T_{e\left(n\right)}\right]}^{2}}{T_{e\left(n-1\right)}}. \end{array}$$

The article "Design and Analysis of Adolescent Physical Health Monitoring System under the Background of Internet of Things and 5G" was retracted in 2023. Reasons: signs of a paper mill; suspected computer-generated content; unreliable results or conclusions; lack of ethics approval or compliance.

#### 2.2.4. Optimal Slot Number Adjustment

Since the label cost is limited by hardware conditions, the number of time slots is not arbitrarily allocated, so the packet is optimized based on label estimation, and the number of time slots is dynamically adjusted based on label estimation to further improve the system throughput in Figure 2.

It can be seen from Figure 2 that the influence trend of throughput change is to increase first and then decrease with the increase of label number. The number of tags corresponding to the number of time slots can be obtained by equation (6), and packet thresholds can also be obtained. The throughput relationship for adjacent time slots can be expressed as

(17) $$\begin{array}{c} S_{1}=S_{2}=\frac{m}{T}\cdot {\left(1-\frac{1}{T}\right)}^{m-1}=\frac{m}{2T}\cdot {\left(1-\frac{1}{2T}\right)}^{m-1}. \end{array}$$

Starting from *T* = 22, the whole number set is successively substituted into equation (17):

(18) $$\begin{array}{c} m=1+\frac{In2}{In\left[\left(2T-1\right)/\left(2T-2\right)\right]}. \end{array}$$

## 3. Design of Physical Health Monitoring System

The integration of the Internet of Things and terrestrial communication network with the 5G mobile communication system as the core is the development trend of the future integrated network of heaven and earth. 5G network has a series of advantages, such as wide coverage, little influence by weather, and strong disaster tolerance. It can provide higher bandwidth when communicating and transmitting data and can meet the design requirements of physical health monitoring system [13].

The article "Design and Analysis of Adolescent Physical Health Monitoring System under the Background of Internet of Things and 5G" was retracted in 2023. Reasons: signs of a paper mill; suspected computer-generated content; unreliable results or conclusions; lack of ethics approval or compliance.

In this chapter, the specific Internet of Things information collection scene is realized based on the ground 5G core network, and the system for monitoring adolescents' physical health is designed. The health and sports information collection is realized by accessing the ground network through 5G network and wearable devices.

### 3.1. Hardware and Software Design of Terminal Node

In this system, the design of sensor acquisition node based on the Internet of Things is the key, which affects the physical health data transmitted through 5G communication technology. Later, the analysis using the client information management system will be performed according to the collected data. Therefore, obtaining correct data plays an important role in the analysis of teenagers' physical health.

#### 3.1.1. Hardware Circuit Design of Acquisition Node

Information collection node is mainly responsible for data collection, including the acquisition and transmission of adolescents' physical health data. The design of the entire collection node is shown in Figure 3.

The sensor module includes sensors and peripheral circuits, and the sensors collect data signals. The power supply circuit supplies power to the whole module.

*(1)Microcontroller Module*. The microcontroller is the core of the collection node [14]. In the collection node, it is responsible for the configuration of sensor parameters, the initialization and operation of protocol stack programs, and the reading and sending of data.

The specific composition of this module is shown in Table 1.

*(2) Acceleration Sensor Module*. The acceleration sensor is used to monitor the acceleration data of teenagers when they move [15]. CC2530 is the main control chip, and the RF transmission circuit is integrated in the chip. The specific structure is shown in Figure 4.

*(3) Temperature Sensor Module*. The temperature sensor node is responsible for detecting the body temperature of teenagers [16], and the specific structure is shown in Figure 5.

#### 3.1.2. Collection Node Hardware Design

The information collection node is responsible for forwarding or receiving data, and its structure is shown in Figure 6.

#### 3.1.3. Program Design of Acquisition Node

The data collected by this node is divided into temperature data and acceleration data so that the system can transmit the movement and temperature data of teenagers in real time.

(1) Acquisition Program of the Acceleration Sensor
    Void UpdateXYZ(void)
    {
    Xaxisl = ReadByte(0 × 32); //Read *x*-axis data
    Xaxish = ReadByte(0 × 33); Yaxisl = ReadByte(0 × 34); //Read *y*-axis data
    Yaxish = ReadByte(0 × 35); Z-axis1 = ReadByte(0 × 36); //Read *z*-axis data
    Zaxish = ReadByte(0 × 37);
    }
Read byte function ReadByte () reads acceleration data stored in three addresses and assigns values to three different variables.
(2) Temperature Sensor Acquisition Program
    For(*i* = 0; *i* < 16; *i*++)
    {
    TMP123_SCK_0();
    TMP123_DELAY();
    TMP123_DELAY();
    TMP123_SCK_1();
    iTmpRead = TMP123_MISO(); iTmpRead<≤1;
    }

According to the acquisition code, the chip line selection is lowered at the beginning of acquisition, and the acquisition data reads the temperature. TMP121 stores temperature data in 16 bits and the temperature values of two bytes are stored separately.

The article "Design and Analysis of Adolescent Physical Health Monitoring System under the Background of Internet of Things and 5G" was retracted in 2023. Reasons: signs of a paper mill; suspected computer-generated content; unreliable results or conclusions; lack of ethics approval or compliance.

### 3.2. Client System Hierarchy

The implementation of the client information management system is shown in Figure 7.

## 4. Experiment

### 4.1. Simulation Analysis of RFID Anticollision Algorithm

In the simulation experiment, the initial number of time slots for each algorithm is 256 by default, and the number of system tags is set to 1500. The number of labels is made from 50 to 1500, the simulation results of each change are recorded, and the simulation results of each change are averaged in order to improve the reliability of data.

#### 4.1.1. Total Time Slot Analysis of System Transmission

This is because the algorithm proposed in this paper is optimized on the previous algorithm, which is more reasonable for grouping, reduces collision slots, and saves the identification time of the RFID system in Figure 8.

#### 4.1.2. System Throughput Analysis

Figure 9 shows that the system throughput rate changes with the increase of the number of tags. When the number of tags exceeds 300, the system throughput of the BEAD algorithm is obviously higher than those of other algorithms. This is due to the reasonable optimization of the number of collision slots in this paper, which estimates of the number of tags more reasonably. When the number of labels to be identified is larger, the throughput curves of the other two algorithms almost coincide and decrease gradually, while the throughput of the BEAD algorithm is stable at over 30%.

Simulation results show that when the number of tags is larger, BEAD algorithm is obviously superior to the other two algorithms, and the BEAD algorithm is more stable. BEAD algorithm has higher system throughput and less communication slot consumption.

### 4.2. Data Acquisition Test

#### 4.2.1. Acceleration Data Acquisition and Test

ADXL345 is a three-axis accelerometer for the *X*-, *Y*-, and *Z*-axes in Figure 10. The corresponding outputs are *X* = 0, *Y* = 0, and *Z* = *g* (where *G* = 9. 8 m/s^2^); in reverse, *X* = 0, *Y* = 0, and *Z* = −1 g (where *G* = 9. 8 m/s^2^).

The article "Design and Analysis of Adolescent Physical Health Monitoring System under the Background of Internet of Things and 5G" was retracted in 2023. Reasons: signs of a paper mill; suspected computer-generated content; unreliable results or conclusions; lack of ethics approval or compliance.

From Figure 10, it is obvious that the *Z*-axis data varies greatly if you move the *Z*-axis vertically upward during running. The *X*-axis and *Y*-axis data change slowly. This feature is in line with the characteristics of human running. The data measured vertically with other axes are the same. When the nodes are mounted in any direction, the measurement data images intersect, but the number change of only one axis is greater than the number change of the other two axes. Experimental results show that the node can work normally.

#### 4.2.2. Temperature Data Acquisition and Test

TMP 121 is selected for the temperature sensor. When the measuring range is −25°C ∼ 85°C, the temperature error reaches 0.5°C, so it can meet the requirements.

The body surface temperature under four steps was detected five times, and the average value was obtained. The measured data are shown in Table 2.

Compared with the actual situation, the measured data accord with the temperature characteristics of the human body surface during movement; and the system is working normally.

### 4.3. Communication Test

This section tests two acquisition nodes and IAR EW C51. Test content is as follows: one node sends data to another node, and LED flashes once after receiving the data. The test steps are as follows:

1. Two nodes are opened, respectively.
2. One node sends data.
3. Another node receives data.
4. LED1 flashes when the data is received.

Table 3 shows the results of the communication distance test.

It can be seen from the table that the normal barrier-free communication distance is about 200 m, and the data reception above 300 m is unstable, but the communication distance of 200 m has met the system requirements.

The power consumption parameters of the test node in normal working state and standby state are shown in Table 4.

It can be seen from the above table that the power consumption of this node is very low.

### 4.4. System Performance Testing

System performance test, also known as a stress test or load test, mainly tests whether the system can work normally under a certain load. The youth performance test for the Internet of Things and 5G background studied in this paper mainly starts with two indicators: user concurrency and response time.

You can choose to set the number of users manually and gradually increase the test index to test the limit of the system. The system for monitoring adolescents' physical health studied in this paper adopts the working state of the system under three conditions: 100 people, 500 people, and 1000 people, and its test results are shown in Table 5.

The article "Design and Analysis of Adolescent Physical Health Monitoring System under the Background of Internet of Things and 5G" was retracted in 2023. Reasons: signs of a paper mill; suspected computer-generated content; unreliable results or conclusions; lack of ethics approval or compliance.

In addition, the system performance tests in different environments are also carried out. The response time in indoor and outdoor environments is given in Figures 11 and 12.

Experiments show that environmental factors have little influence on the response time and accuracy of the system. With the help of the proposed system, the physical health status of teenagers can be monitored in real time. This system is helpful to the healthy management of teenagers' physique and has high popularization and use value.

## 5. Conclusions

This paper mainly completes the design and analysis of systems monitoring adolescents' physical health under the background of Internet of Things and 5G and realizes data collection and 5G communication transmission; the visual display, storage, and management of health and exercise information are completed. Teenagers' physical health data are collected through wearable devices based on the Internet of Things, and then data is sent to the intelligent terminals or servers by using Internet of Things information collection based on ground 5G core network, and then the intelligent terminals or servers process teenagers' physical health data in real time to analyze their physical health. This system can be used to detect the physical health information of teenagers in real time, and, according to the quantified health level and exercise amount, it can achieve the purpose of monitoring teenagers' physical health.

## Figures and Tables

**Figure 1:** Schematic diagram of such area grouping.

**Figure 2:** Throughput under different fixed slot numbers.

**Figure 3:** Block diagram of acquisition node.

**Figure 4:** Block diagram of the acceleration sensor module.

**Figure 5:** Block diagram of the temperature sensor module.

**Figure 6:** Block diagram of coordinator composition structure.

**Figure 7:** Hierarchical structure of this information system.

**Figure 8:** Comparison of total time slots.

**Figure 9:** Throughput comparison.

**Figure 10:** Acceleration-time curve (*Z*-axis).

**Figure 11:** Response time of the device in an indoor environment.

**Figure 12:** Response time of the device in an outdoor environment.

**Table 1:** Comparison table between sensor floor and I/O interface.

External sensor, power supply	CC2530 pins
BUTTON1	P0.1
ADXL_MISO	P0.2
ADXL_MOSI	P0.3
ADXL_CSN	P0.4
ADXL_SCLK	P0.5
INT1	P0.6
TMP_DATA	P0.7
INT2	P2.0
LED1	P1.0
LED2	P1.1
TMP_CS	P1.3
DEBUG_CSN	P1.4
DEBUG_SCLK	P1.5
DEBUG_MOSI	P1.6
DEBUG_MISO	P1.7
DEBUG_DD	P2.1
DEBUG_DC	P2.2
RESET	RESET_N

The article "Design and Analysis of Adolescent Physical Health Monitoring System under the Background of Internet of Things and 5G" was retracted in 2023. Reasons: signs of a paper mill; suspected computer-generated content; unreliable results or conclusions; lack of ethics approval or compliance.

**Table 2:** Temperature acquisition data.

Step number	1 time	2 times	3 times	4 times	5 times	Mean value
93 steps	27.1	27.8	27.5	28.7	28.1	27.6
110 steps	28.4	27.5	28.8	29.5	28.8	28.3
159 steps	31.9	30.9	30.7	31.5	31.6	31.4
180 steps	32.1	32.5	32.3	32.4	32.2	32.6

**Table 3:** Communication distance test.

Test distance	10m	50 m	100 m	150 m	200 m	320 m	340 m
Reception	Normal	Normal	Normal	Normal	Normal	Unstable	Unable to receive

**Table 4:** Node power consumption test.

Maximum emission current (mA)	Maximum current received (mA)	Operating voltage	System power consumption	Transmit power consumption	Standby working current
29	24	3.1 V∼3.6 V	89.9∼104.4 mW	≤105 mW	＜0.2 mA

**Table 5:** Performance test results of a system monitoring adolescents' physical health based on 5G and Internet of Things information collection.

Number of users	Average response time (ms)	Peak response time	Test conclusion
100	0.915	1.155	Pass
500	1.223	1.853	Pass
1000	2.456	2.876	Pass

## Data Availability

The experimental data used to support the findings of this study are available from the corresponding author upon request.
